The article "Cases of Ultrasound-Diagnosed Right Aortic Arch with Right Arterial Duct and the Treatment" was retracted in 2022. Reason: concerns about the peer review.

# Cases of Ultrasound-Diagnosed Right Aortic Arch with Right Arterial Duct and the Treatment

**DOI:** 10.1155/2022/8252808

**Published:** 2022-01-28

**Authors:** Xu Li, Luo Jiamin, Wang Junmei

**Affiliations:** Department of Ultrasound, Women's Hospital, School of Medicine, Zhejiang University, Hangzhou, Zhejiang Province, China

## Abstract

This paper aims to discuss the value of ultrasound to diagnose right aortic arch with right arterial duct. A retrospective analysis of fetal echocardiography characteristics of 10 fetuses who were diagnosed as right aortic arch with right arterial duct from December 2016 to March 2021 is made, and focus is put on the relationship between the aortic arch and arterial duct, and the position of aortic arch, arterial duct arch and trachea on the three vessels and trachea view (3VT). As a result, all 10 cases with right aortic arch and right arterial duct do not show aberrant left subclavian artery, and aortic arch with arterial duct are still connected as “V-shaped”, and do not get vascular rings. In conclusion, 3VT can simply and clearly detect the right aortic arch, and the key to diagnosing the right aortic arch and right arterial duct is thorough inspection of the aortic arch, arterial duct, and trachea in their respective positions.

## 1. Introduction

As for a healthy person, the aortic arch is on the left of the trachea. As the aorta goes down the right side of the main bronchus, it is referred as right aortic arch (RAA), and the occurrence rate is about 1‰ [1]. Right aortic arch is generally divided into 2 types: right aortic arch with aberrant left subclavian artery (RAA-ALSA) and right aortic arch with mirror image branching (RAA-MB). RAA-ALSA and left arterial duct are the most common vascular ring malformations, whereas right aortic arch accompanied by right arterial duct will not form effective vascular rings or cause compression to the trachea and esophagus due to the reason that both aortic arch and arterial duct are on the right side of the trachea. This paper aims to explore the characteristics of prenatal echocardiography of right aortic arch and right arterial duct and the treatment.

## 2. Data and Method

### 2.1. Research Object

Ten babies identified with right aortic arch with right arterial duct using prenatal echocardiography in our institution between December 2016 and March 2021 were selected as study participants. They are all monocyesis, and their ages vary from 25 to 46 years, with an average of 31.8 + 6.1 years, and their gestation periods span from 22 to 32 weeks, with an average of 25.5 + 2.7 weeks.

### 2.2. Instrument and Method

GE VolusionE8, E10 and Samsung WS80A color Doppler ultrasound diagnostic apparatus with a probe frequency of 2 ~ 8 MHz are used in the research. With the condition for the fetus heart examination in middle-late pregnancy, the echocardiography of sections is performed in accordance with ISUOG guidelines. Determine fetal direction, left or right, fetal viscera relation and heart location. Standard ultrasound sections of fetal heart: including upper abdominal transverse section, four-chamber cardiac section, left and right ventricular outflow tract section, the aortic arch section, arterial duct section, three vessel view(3VV), grayscale and color Doppler flow imaging of three vessel and trachea view (3VT) with the fetus echocardiography. While there is a doubt about the position of the aortic arch and arterial duct we especially observe the connection status of the aortic arch and pulmonary arterial duct, and the relative position of the aortic arch, arterial duct and trachea. The location of the aortic arch in fetal heart and its abnormal diagnosis are determined by two experienced physicians.

The article "Cases of Ultrasound-Diagnosed Right Aortic Arch with Right Arterial Duct and the Treatment" was retracted in 2022. Reason: concerns about the peer review.

### 2.3. Follow-Up of Cases

As for fetuses diagnosed as right aortic arch and right arterial duct according to prenatal ultrasound, a comprehensive evaluation of the risk of pregnancy is made to decide whether to terminate pregnancy or not based on the analysis of other possible malformations and chromosomal karyotype. Ultrasound examinations of newborn babies are made to compare the results with that of the antenatal period.

## 3. Result

As illustrated in Table 1, five of the ten instances include foetuses with a straight right aortic arch and a right arterial duct, and one involves a transposition of the major arteries. 1 instance has a ventricular septal defect in addition to an aortic saddle, 1 case is complicated by PRUV (Persistent Right Umbilical Vein), 1 case has lateral ventricular widening without evidence of gallbladder, and 1 case has bilateral hydronephrosis. None of these 10 cases has the aberrant left subclavian artery in the right aortic arch and right arterial duct, and thus no vascular rings are formed.

5 cases of sheer right aortic arch with right arterial duct, 1 case accompanied by PRUV, 1 case of bilateral hydronephrosis are confirmed generally in good condition by neonatal echocardiographies, whereas the case of broadening lateral ventricle, with no obvious gallbladder is found with ASD (atrial septal defect), congenital tracheal deformity, deafness, cryptorchidism and some other malformations after birth. Postpartum whole-exon genetic testing shows that CHD7 gene mutates and presents as CHARGE syndrome and Kallmann syndrome V. In the other 2 cases, pregnant women and their family choose odinopoeia and refuse to perform autopsies.

The article "Cases of Ultrasound-Diagnosed Right Aortic Arch with Right Arterial Duct and the Treatment" was retracted in 2022. Reason: concerns about the peer review.

The echocardiography of the fetal of right aortic arch with right arterial duct shows that both the aortic arch and arterial duct are on the right of trachea, not as “U-shaped” but as “V-shaped”, as shown in Figure 1.

## 4. Discussion

Normally, the left aortic arch evolves from the 4th left arch artery and the left dorsal aorta, while the right side degenerates. If the right side of the 4th pair of arcuate arteries does not degenerate and the left side degenerates, the right aortic arch will occur [2]. Vascular rings are congenital aortic arch and branching vascular malformations, which wrap around and compress the trachea and esophagus. Vascular rings can wrap the trachea and esophagus, completely or partially. The severity of clinical symptoms such as dyspnea in trachea and esophagus or dysphagia in patients with compression of trachea and esophagus depends on how tight Vascular rings surround and compress the trachea and esophagus. Without other cardiovascular malformations, i.e., normal circulatory physiology, vascular rings will not cause significant changes in each atrioventricular cavity. Among all the malformations, the right aortic arch accompanied by left aberrant subclavian artery and left arterial duct are the most common seen. Since the normal ascending aorta continues to the right aortic arch and descending aorta, and the left aberrant subclavian artery arises from the upper part of the right descending aorta, and the right subclavian artery starts from the distal end of the right subclavian artery, and ran along the left side of the esophagus, the left aberrant subclavian artery is also called the left subclavian artery of the back esophagus.

Right aortic arch, the left aberrant subclavian artery and arterial duct appear “U-shaped” arterial arch on the left of trachea and esophagus and surround them. Double aortic arch is commonly seen in vascular rings. The position of ascending aorta shows normal and can be divided into left and right aortic arches in front of the trachea. In trachea, the right aortic arch is usually slightly higher than the left, which passes the trachea and esophagus and into the descending aorta, and then meets the left arch, together making an “O-shaped” aortic ring that surrounds trachea and esophagus. The two fetuses of right aortic arch with left arterial duct, and the right aberrant subclavian artery will see a relatively good prognosis in that they may geta slight trachea & esophagus compression after birth, but they will find a gasping, a recurrent respiratory infection, or even difficulty in swallowing, and will have to receive a surgical treatment after birth due to trachea compression caused by double aortic arch and pulmonary artery sling.

The article "Cases of Ultrasound-Diagnosed Right Aortic Arch with Right Arterial Duct and the Treatment" was retracted in 2022. Reason: concerns about the peer review.

According to documents [3], individuals with straight right aortic arch and right arterial duct had a favourable prognosis. Certain children with a right aortic arch and a left arterial duct may need trachea compression and, in rare situations, surgery. According to certain domestic researchers [4], a baby with RAA but no additional intracardiac anomalies or chromosomal disorders may have a favourable prognosis. The prognosis of a foetus complicated by cardiovascular abnormalities is severity dependent. Two examples of odinopoeia are discussed in this article, both of which include the fusion of additional intracardiac abnormalities. Five of the eight living instances had a sheer right aortic arch with a right artery duct, and two cases have a combination of non-complex cardiac structural anomalies., Among the youngsters being monitored, the oldest is three years old and in excellent health. According to the record, one prenatal diagnostic demonstrates lateral ventricle widening without the presence of a gallbladder. Now sixteen months old, the kid is diagnosed with postpartum ASD, congenital tracheal deformity, deafness, cryptorchidism, and other abnormalities. The whole gene exon test performed after delivery reveals that a CHD7 gene mutation occurs, which is defined by CHARGE syndrome and Kallmann syndrome type 5. Two instances undergo prenatal amniotic fluid puncture, and the results indicate that the chromosomal karyotype is normal. A cord blood sample is obtained in one example, and the chromosomal karyotype is normal., Antenatal detection of fetal RAA shall be done only after effectively communicating with the pregnant mother and her family. Most fetuses with pure RAA can get a good prognosis, and thus odinopoeia should not be abused. Fetal with right aorta and intracardiac abnormalities should get chromosome karyotype and gene sequence examinations [5]. Documents show that after birth, the rate of right aortic arch accompanied by 22q11.2 copy number variations (CNVs) ranges from 9% to 12% [6, 7] (right arch cases), risk of antenatal sheer right aortic arch with 22q11.2 CNVs is 5.1% (95% CI, 2.4% ~8.6%) [8]. Peng Ruan et al. [9], observe that 5% fetuses suffer from right aortic arch with 22q11.2 CNVs. Therefore, when right aortic arch is found in ultrasound test, chromosomal microarray analysis (CMA) should be made to detect and exclude chromosomal abnormalities. Tetralogy of fallot is the most common intracardiac anomaly type of fetuses with right aortic arch. The occurrence of combination of intracardiac and extracardiac abnormalities may affect the prognosis of fetal with right aortic arch.

The article "Cases of Ultrasound-Diagnosed Right Aortic Arch with Right Arterial Duct and the Treatment" was retracted in 2022. Reason: concerns about the peer review.

Left or right aortic arch is determined by the aortic arch and trachea location. RAA occurs when the aortic arch is located to the right of the trachea. The 3VT section clearly demonstrates the aortic arch and trachea's positional connection, making it a sensitive and effective way for ultrasonic diagnosis of RAA [10], and the efficacy of ultrasonic diagnosis of foetal RAA by 3VT has been well acknowledged [11–13]. Because aortic arch with left artery duct is more prevalent than aortic arch with no left arterial duct, a “U-shaped” link is often found in 3VT. However, there is no “U-shaped” connection in the case of the right arterial duct, which makes it simple to misdiagnose or neglect [14]. As a result, the aortic arch and trachea location connection should be carefully studied on the three-vessel trachea segment. As long as the aortic arch is on the right, the condition is classified as right aortic arch. After that, determine if the arterial duct is located on the right or left side of the trachea. The fetus with right aortic arch and arterial duct may sometimes combine a left aberrant subclavian artery and thus may also have the “U-shaped” vascular rings [15–17]. However, it is difficult to determine the occurrence of the left aberrant subclavian artery through a three-vessel tracheotomy because it needs the confirmation of a coronary section.

To summarise, 3VT is the primary portion for diagnosing foetal RAA. The key to identifying right aortic arch with right arterial duct is to carefully observe the connection of the aortic arch, arterial duct, and trachea in terms of location. While RAA is detected during prenatal screening, a complete diagnosis and observation of whether intracardiac or cardiac complications occur should be performed to give more comprehensive and accurate information for perinatal counselling and prompt postpartum therapy.

## Figures and Tables

**Figure 1:** 3VT ultrasound imaging of fetuses suffering from right aortic arch accompanied with right arterial duct shows that both the aortic arch and arterial duct are on the right of trachea. (LPA: left pulmonary artery, T: trachea, DA: arterial duct, AO: the aortic arch).

**Table 1:** Antenatal diagnosis and postpartum follow-up results in 10 fetuses.

Number	Gender	Other intracardiac and extracardiac abnormalities (antenatal)	Related genetic test (antenatal)	Other intracardiac and extracardiac abnormalities (postpartum)	Prognosis	Postpartum ultrasound result	Remarks
1	—	Corrected transposition of great arteries	Amniocentesis: Normal karyotype	—	26 weeks before odinopoeia	—	Autopsy: Refused
2	—	Ventricular septal defect, aortic saddle		—	28 weeks before odinopoeia	—	Autopsy: Refused
3	Male	Lateral ventricle widened, gallbladder not shown	Umbilical blood puncture: Normal chromosome karyotype	ASD, congenital tracheal malformation, deafness, cryptorchidism and other malformations	40 weeks before eutocia	Proved	CHD7 gene mutates
4	Male	Double kidney seeper	—	—	39 weeks before eutocia	Proved	
5	Male	—	—	ASD	37 weeks before cesarean section	Proved	
6	Female	PRUV	Amniocentesis: Normal karyotype	PRUV	40 weeks before cesarean section	Proved	
7	Male	—	—	—	40 weeks before eutocia	Proved	
8	Female	—	—	—	38 weeks before eutocia	Proved	
9	Female	—	—	—	39 weeks before cesarean section	Proved	
10	Male	—	—	—	38 weeks before eutocia	Proved	

The article "Cases of Ultrasound-Diagnosed Right Aortic Arch with Right Arterial Duct and the Treatment" was retracted in 2022. Reason: concerns about the peer review.

## Data Availability

The data used to support the findings of this study are included within the article.
